The article "CT Image Changes of Severe Acute Pancreatitis Based on Smart Electronic Medical Augmented Reality in Nursing Practice" was retracted in 2023. Reasons: signs of a paper mill; suspected computer-generated content; unreliable results or conclusions; lack of ethics approval or compliance.

# CT Image Changes of Severe Acute Pancreatitis Based on Smart Electronic Medical Augmented Reality in Nursing Practice

**DOI:** 10.1155/2021/5522492

**Published:** 2021-04-26

**Authors:** Defen Zhang, Shifang Mao, Siyou Lan, Chengli Zhou, Xiaoyan Liu

**Affiliations:** ^1^Emergency Intensive Care Unit, The Affiliated Hospital of Southwest Medical University, Luzhou 646000, Sichuan, China; ^2^Department 1 of Respiratory and Critical Diseases, The Affiliated Hospital of Southwest Medical University, Luzhou 646000, Sichuan, China

## Abstract

Severe acute pancreatitis (SAP) is traditionally treated with chemical analysis. Faced with the increasing maturity of CT imaging technology, it is necessary to use more advantageous CT imaging to treat SAP. In this article, 72 SAP patients admitted to the Affiliated Hospital of Southwest Medical University were selected for study, of which 62 were severely ill, 8 were exacerbated, and 2 changed from severe to mild. This article combines the patient's case records and related CT images during treatment from the perspective of nursing and conducts nursing research on the application of CT image changes in severe acute pancreatitis in nursing practice. CT image processing uses CT imaging system workstation (DICOM). The results of the study showed that, in the care of patients, 21 cases had recurrence after internal drainage, and the cure rate was 91.1%. Internal drainage is an effective way to treat SAP. The higher the incidence of pancreatitis, the more likely it is to relapse after SAP internal drainage, which may be related to repeated episodes of pancreatitis and repeated inflammation of the pancreas and pancreatic duct damage. 4 of the relapsed cases in this article are postchronic pancreatitis SAP, and the relapsed cases account for 50% of the chronic pancreatic cases. This may be due to chronic fibrosis of the branched and main pancreatic ducts, continuous abnormal pancreatic juice drainage. Therefore, it is necessary to further explore the prognosis of different causes of SAP. In terms of complication care, the overall complication rate was 16.6%. One patient died of postoperative hemorrhage. Analysis of the causes of cyst recurrence and complications may be closely related to the mechanism of the occurrence and development of SAP. The initiating factor of SAP is that the pancreatic tissue is damaged due to inflammation, trauma, or microcirculation disorder, and then the pancreatic juice leaks out of the pancreas, wrapping the pancreatic juice; it takes a certain time for the capsule of fibrous knot tissue to form and strengthen.

## 1. Introduction

Severe acute pancreatitis (SAP) is a disease with a high mortality rate and a rapid onset. There are still some problems in nursing. For the diagnosis and nursing of SAP, there are two diagnostic models that are generally recognized: one is the Japanese model and the other is the American model. These two models carry out modeling research on the serum condition of SAP. And other related organs are also involved.

The article "CT Image Changes of Severe Acute Pancreatitis Based on Smart Electronic Medical Augmented Reality in Nursing Practice" was retracted in 2023. Reasons: signs of a paper mill; suspected computer-generated content; unreliable results or conclusions; lack of ethics approval or compliance.

Siegel et al. set serum IgG4 level, CT image of pancreas, and endoscopic cholangiopancreatography as observation indexes, and its CT positive manifestations were low-density shadow around pancreas, delayed enhancement, and atrophy of pancreatic body and tail; pancreaticocholangiography showed inhomogeneous and diffuse pancreatic duct stenosis, nondilation of main pancreatic duct, and stenosis of secondary pancreatic duct [1]. Riker et al. distinguished SAP based on CT findings, serum IgG4 level, and other organ involvement. If the diagnosis cannot be confirmed, tissue biopsy or hormone therapy is recommended [2]. Deshpande et al. differentiated pancreatic cancer and SAP according to serum IgG4 level combined with CA-199 level. The results showed that serum IgG4 level was more than 2 times higher than the normal value and serum CA-199 level was lower than 85 U/ml, which were important diagnostic indicators for distinguishing sap from pancreatic cancer [3]. Kamisawa et al.'s study pointed out that patients with mild elevated serum IgG4 should be treated with caution, and excessive dependence on serum IgG4 as a diagnostic marker of SAP may lead to missed diagnosis of pancreatic tumor [4]. In Chari et al.'s study, there were 22 patients with pancreatic tumor whose serum IgG4 was higher than 1.35 g/L, and the median value was 2.49 g/L. Among them, there were 8 patients whose serum IgG4 was more than 2 times higher than the normal value [5].

He et al. pointed out that serum IgG4 more than 2 times the normal value can improve the specificity of diagnosis of SAP [6]. However, in Okazaki et al. study, only one patient was diagnosed as pancreatic cancer with SAP, and the serum IgG4 value was 9.33 g/L [7]. Hamano et al. believed that if the serum IgG4 level in patients with obstructive jaundice is increased, even if it is more than 2 times of the normal value, the possibility of the malignant tumor cannot be ruled out in the absence of other organ involvement, and tissue biopsy is feasible to identify malignant tumor [8]. Choi et al.'s study showed that simple serum IgG4 was 2 times higher than the normal value, which could not differentiate sap from pancreatic cancer [9]. Okazaki et al. analyzed that 10.1% of 548 patients with pancreatic cancer had elevated serum IgG4 but did not find the significance of elevated serum IgG4 on the prognosis of pancreatic cancer [10]. The above studies mainly analyze the physiological pathology of pancreatitis from the perspective of serum, but for severe acute pancreatitis, the effect is very slow from the chemical point of view, so it is necessary to treat patients in a faster way, and CT imaging technology can solve the above problems to a great extent.

The article "CT Image Changes of Severe Acute Pancreatitis Based on Smart Electronic Medical Augmented Reality in Nursing Practice" was retracted in 2023. Reasons: signs of a paper mill; suspected computer-generated content; unreliable results or conclusions; lack of ethics approval or compliance.

This article first constructed a DICOM 3D model of the distal pancreas and then selected the reference point of the CT image to analyze the image and finally analyzed the application of the CT image changes of severe acute pancreatitis in nursing practice. In this article, 72 SAP patients admitted to the Affiliated Hospital of Southwest Medical University were selected as the research object. Among them, 62 were severely ill, 8 were deteriorating, and 2 had changed from severe to mild symptoms. This article combines the patient's case records during treatment and related CT images to study the application of CT image changes in severe acute pancreatitis in nursing practice. CT image processing uses CT imaging system workstation (DICOM).

## 2. Severe Acute Pancreatitis and CT Imaging Technology

### 2.1. Symptoms and Conventional Treatment of Severe Acute Pancreatitis (SAP)

At present, there is no uniform standard for the image acquisition methods and preoperative pancreatic planning methods required for pancreatic guide plate preparation [11, 12]. Although the accuracy of CT scan in cartilage display and reconstruction model is not as good as MRI, and the articular surface cannot be used as a reference, the model surface based on CT image reconstruction is smoother and flat, which is more accurate than MRI as a positioning reference [13, 14]. There are also studies on the construction of a pancreatic model based on CT images, but the pancreas is still based on the subchondral bone. During the operation, the articular cartilage and marginal osteophytes need to be divided for the placement of the pancreatic guide plate [15–17]. However, the subchondral bone that cannot be controlled when biting the articular cartilage is the same or similar to the preoperative plan, and the human error is large. In the prolonged development stage of SAP, the islet cells have not yet completely failed, and the coexistence of impaired insulin secretion and insulin resistance is the cause of glucose metabolism disorders. At this time, treatment from multiple aspects is often more effective [18]. The treatment methods are becoming more abundant, puncture drainage is convenient and economical, but the incidence of complications is high; endoscopic technology has obvious advantages, but the secondary treatment rate is higher; the open drainage is classic and the curative effect is stable. Recently, there have also been reports of internal drainage surgery in SAP assisted by Da Vinci robot [19]. Regardless of the method, the basic principle of its treatment is mainly to deal with abnormal drainage of pancreatic juice. The location and size of the cyst, the general state of the patient, and comorbidities should be considered in the clinical management of SAP. Choose the treatment plan that benefits the patient the most [20]. Therefore, the early diagnosis of pancreatic cancer is a challenge for abdominal surgeons challenge for abdominal surgeons. Early detection of tumors is one of the keys to successful treatment. The identification of pancreatic cancer is also crucial to the effectiveness of treatment. Abdominal images of most patients with pancreatic tumors suggest that the pancreas occupies a space, but it is often difficult to distinguish between benign and malignant. With the continuous development of medicine, autoimmune pancreatitis (AP) has gradually been recognized. The increase in serum IgG4 level more than twice the normal value is considered an important diagnostic indicator for type I SAP. However, there are also a small number of pancreatic cancer patients. Serum IgG4 is elevated, but the elevated level usually does not exceed 2 times the normal value [21]. Clinically, SAP and pancreatic head tumors have many common features, including painless jaundice, new-onset diabetes, and weight loss [22]. Therefore, distinguishing between SAP and pancreatic cancer is still challenging for abdominal surgeons [23–25]. Due to the damage of SAP to acinar cells, it may cause multiple organ dysfunction syndrome (MODS) in the acute phase of the disease. In the middle and late stages of the disease, the translocation of intestinal bacteria causes extrapancreatic tissue infection (EPI) [26]. EPI is a common SAP complication, including pancreatic infection, urinary system infection and bacteremia, etc., which have a serious adverse effect on the prognosis of patients. Especially for patients with severe pancreatitis (SAP), the incidence of EPI is higher than 50%, but the change of the body's immune function is the basis of the occurrence and pathological progress of SAP [27]. In addition, SAP may cause a significant increase in the level of systemic inflammatory response markers, and whether these easily available clinical indicators can be used in the diagnosis of secondary pancreatic infection in SAP patients remains to be studied [28].

The article "CT Image Changes of Severe Acute Pancreatitis Based on Smart Electronic Medical Augmented Reality in Nursing Practice" was retracted in 2023. Reasons: signs of a paper mill; suspected computer-generated content; unreliable results or conclusions; lack of ethics approval or compliance.

### 2.2. CT Image Model of Augmented Reality Based on Smart Electronic Medical DNN

For the contradiction between the depth and performance degradation of CT image classification network of severe acute pancreatitis, the residual structure is used:

(1) $$\begin{array}{c} 2\text{DConv}=\frac{n\sum_{i=1}^{n}\sum_{j=1}^{n}w_{ij}\left(x_{i}-\bar{x}\right)\left(xj-\bar{x}\right)}{\sum_{i=1}^{n}\sum_{j=1}^{n}w_{ij}{\left(xi-\bar{x}\right)}^{2}}=\frac{n\sum_{i=1}^{n}\sum_{i\neq j}^{n}w_{ij}\left(x_{i}-\bar{x}\right)\left(xj-\bar{x}\right)}{S^{2}\sum_{i=1}^{n}\sum_{j=1}^{n}w_{ij}}. \end{array}$$

It consists of two parts: the first part is the identity mapping; the second part is bottleneck structure, that is, first through a 2dconv with 1 × 1 convolution kernel, then through a 2dconv with 3 × 3 convolution kernel, and then through a 2dconv with 1 × 1 convolution kernel. At the same time, BN operation and relu operation are performed between different convolution operations [29, 30]. For the contradiction between CT image resolution and receptive field of severe acute pancreatitis, this algorithm designs an expanded residual structure, as shown in equation (2).

(2) $$\begin{array}{c} {\text{SC}}_{\text{CT}}=\frac{\sum_{j=1}^{k}\sum_{h=1}^{k}\sum_{t=1}^{n_{j}}\sum_{r=1}^{n_{h}}\left|y_{ij}-y_{hr}\right|}{2n^{2}u}. \end{array}$$

Different from the residual structure, by adding 3 ∗ 3 expansion convolution, the larger receptive field is successfully modeled, and the defect of single receptive field is solved to a certain extent. In order to improve the detection sensitivity of electrochemistry, the electrode fixed CT image boundary complex can be rolled

(3) $$\begin{array}{c} u_{h}\leq u_{j}\leq ...\leq u_{k}, \end{array}$$

(4) $$\begin{array}{c} G=G_{w}+G_{nb}+G_{t}, \end{array}$$

(5) $$\begin{array}{c} P\left(d_{i},w_{j}\right)=P\left(d_{i}\right)P\left(w_{j}|d_{i}\right);P\left(w_{j}|d_{i}\right)=\sum_{k=1}^{K}P\left(w_{j}|z_{k}\right)P\left(z_{k}|d_{i}\right). \end{array}$$

In the channel attention module, focus on the weight distribution of different channels, input *h*h × *w* × *C* conv4_ *x*. After avgpool (average pooling) and maxpool (maximum pooling); the size is converted to 1 × 1 × C. Considering the need to make full use of the different information obtained by the two pooling operations, MLP (multilayer perceptron) with shared parameters is added [31]. Then, the scaling factor is obtained by activating function *σ*. Finally, it is compared with the initial CT image feature map conv4 of severe acute pancreatitis_ spatial attention module focuses on the weight distribution of spatial information

(6) $$\begin{array}{c} {\text{MLP}}_{jh}=\frac{\sum_{Z=1}^{h_{j}}\sum_{r=1}^{n_{h}}\left|y_{ji}-y_{hr}\right|}{n_{j}n_{h}\left(u_{j}+u_{h}\right)}, \end{array}$$

(7) $$\begin{array}{c} l_{\text{ssim}}=1-\frac{\left(2\mu_{x}\mu_{y}+C_{1}\right)\left(2\sigma_{xy}+C_{2}\right)}{\left(\mu_{x}^{2}+\mu_{y}^{2}+C_{1}\right)\left(\sigma_{x}^{2}+\sigma_{y}^{2}+C_{2}\right)}, \end{array}$$

(8) $$\begin{array}{c} G_{t}=\sum_{j=2}^{k}\sum_{h=1}^{j-1}G_{jh}\left(p_{j}s_{h}+p_{h}s_{j}\right)D_{jh}\left(1-D_{jh}\right). \end{array}$$

The modeling process of S (a) module in amdrc net is divided into five stages, and the final CT image features of severe acute pancreatitis are classified into three levels. The classifier uses softmax loss, which is essentially: transform the new CT image into log likelihood in probability space:

(9) $$\begin{array}{c} {℘}_{\kappa }=\frac{2k}{k+1}+\left[\frac{1}{2}+\frac{1}{2k}\right]{\left[\frac{c_{2}-c_{1}}{3}\right]}^{2}+\frac{2\left(c_{2}-c_{1}\right)}{3}, \end{array}$$

(10) $$\begin{array}{c} d_{jh}=\int_{0}^{\infty }\text{d}F_{j}\left(y\right)\int_{0}^{y}\left(y-x\right)\text{d}F_{h}\left(x\right), \end{array}$$

(11) $$\begin{array}{c} \ln\text{ softm}ax_{it}=a_{0}+a_{1}du\;*dt+\sum_{i=1}^{N}b_{j}Xu+\varepsilon_{u}. \end{array}$$

The loss value is minimized by forward propagation and back propagation. The softmax loss function can effectively distinguish the differences between classifications and provide nonlinear expression capability for the network. At this time, softmax normalizes the n-dimensional vector (*n* = 3) output from the full connection layer (the sum of all dimension values is 1), and the values in the n-dimensional vector represent the probability value of the prediction tag, respectively. The specific calculation process is shown in (12):

(12) $$\begin{array}{c} k_{t1}\left[i\right]=\sum_{j}\cos\left(w_{i}^{1},w_{j}^{2}\right), \end{array}$$

(13) $$\begin{array}{c} \text{LS}\left(x\right)=\frac{1}{\sqrt{2\pi }}\exp\left(-\frac{x^{2}}{2}\right), \end{array}$$

(14) $$\begin{array}{c} \text{HT}=\tanh\left(w_{c}x_{t}+u_{c}\left(r_{t}\Theta h_{t-1}\right)+\text{BC}\right)+C, \end{array}$$

(15) $$\begin{array}{c} h_{t}=z_{t}\Theta h_{t-1}+\left(1-z_{t}\right)\Theta h_{t}+W. \end{array}$$

In the expression, LS represents the loss function of gradient descent for softmax results, *X* represents the total input training data, BC represents the input data, HT represents the category of CT image of severe acute pancreatitis, *C* represents the total category of training data, and W represents the parameters of network model training and learning. Using LiFePO_4_ as a signal probe can not only expand the application of lithium-ion battery materials, but also expand the application of biosensors:

(16) $$\begin{array}{c} \sigma t=\frac{\sqrt{\left(1/n\right)\sum_{i=1}^{n}{\left({\text{FI}}_{it}-{\text{FI}}_{it}\right)}^{2}}}{{\text{FI}}_{it}}, \end{array}$$

(17) $$\begin{array}{c} u_{\left(j/i\right)}=w_{ij}A_{i}, \end{array}$$

(18) $$\begin{array}{c} x_{H}=\frac{p_{2}-p_{1}+1}{2}. \end{array}$$

Finally, the self-attention module network provides a new function for long-distance modeling of CT images of coronal pancreatitis. The calculation process is as follows:

(19) $$\begin{array}{c} \ln\left(\frac{{\text{FI}}_{it}}{{\text{FI}}_{it}-1}\right)=\alpha +\beta \;\ln\;FI_{it}-1+v_{i}+{ℑ}_{t}, \end{array}$$

(20) $$\begin{array}{c} \psi =\sum_{x=1}^{\theta }Vx=\sum_{x=1}^{\vartheta }\left(\frac{Wx}{\sum_{1}^{n}W_{ℑ}}Sx\right). \end{array}$$

Although CT can well identify ischemic lesions, it is difficult to show quite a few ischemic lesions on CT in the early stage of the disease due to different degrees of ischemia. CT perfusion imaging is an examination method to judge the blood flow status of ischemic lesions. The blood flow status of pancreas can be observed by injecting a contrast agent [32].

The article "CT Image Changes of Severe Acute Pancreatitis Based on Smart Electronic Medical Augmented Reality in Nursing Practice" was retracted in 2023. Reasons: signs of a paper mill; suspected computer-generated content; unreliable results or conclusions; lack of ethics approval or compliance.

## 3. Design of CT Image Changes of Severe Acute Pancreatitis in Nursing Practice

### 3.1. Samples

This article selects 72 SAP patients admitted to the Affiliated Hospital of Southwest Medical University as the research object, 62 of which are severe, 8 are deteriorating, and 2 have changed from severe to mild symptoms. This article combines the patient's case records during treatment and related CT images to study the application of CT image changes in severe acute pancreatitis in nursing practice. CT image processing uses the CT imaging system workstation (DICOM) for research. This software (Made in China) only exports images. The other functions and safety of this software have not been involved.

### 3.2. Sample Processing and Analysis Methods

#### 3.2.1. Construction of Three-Dimensional Model of Distal Pancreas in DICOM

DICOM is based on the formation of “Mask” on two-dimensional CT images. The software has several image features, but it can only segment areas where the thresholds are clearly different. First of all, the pancreatic CT image of patients with pancreatic osteoarthritis will show edge defect by software automatic segmentation, especially when the scanning current parameters are not fixed, and the difference of osteophyte edge display is obvious; the larger the scanning current is, the clearer the osteophyte display is, but the patient's radiation is increased; the scanning current is too small, the worse the osteophyte display is, so manual repair is often needed; however, when the software is used to customize, if the threshold is too large, the incomplete the “Mask” edge is, the worse the division of osteophytes is, and the reconstructed model is incomplete after using the “calculate 3D” function in the software; if the threshold is too small, the rougher the “Mask” edge is, the lower the recognition degree of the edge is, resulting in the rougher edge of the reconstructed model and the appearance of redundant “spike.” Secondly, when manually editing the “Mask,” it is often necessary to process the coronal, sagittal, and cross-sectional images at the same time. Since the recognition of the displayed image of the osteophyte differs from person to person in three stages, the shape of the reconstructed 3D model also differs. During this study, the CT scan parameter of the pancreas was 1 mm thick, which could better indicate the condition of the pancreatic marginal osteophytes within the structure, which would help to accurately reconstruct the pancreatic bone model.

The article "CT Image Changes of Severe Acute Pancreatitis Based on Smart Electronic Medical Augmented Reality in Nursing Practice" was retracted in 2023. Reasons: signs of a paper mill; suspected computer-generated content; unreliable results or conclusions; lack of ethics approval or compliance.

#### 3.2.2. Selection of Reference Points for CT Image Location

In this paper, we selected the anterior cortex of the pancreas and the osteophytes at the edge of the medial and lateral condyles as the reference points and confirmed that the anterior cortex of the pancreas has the greatest reference value through intraoperative observation. The goodness of fit of the pancreatic guide plate on the CT image directly affects the position of the entire pancreatic interface and also the force line of the pancreas. However, only anterior pancreatic reference can provide CT images of the stability of the pancreatic guide plate located distal to the pancreas. It is necessary to increase the osteophyte at the edge of the medial and lateral condyles of the pancreas as a fixed reference, and it can also be used as a reference interface for pancreatic surgery through the condyle axis, so as to view the rotation force line more intuitively during the operation. In conclusion, CT image preparation based on pancreatic CT and lower extremity full-length weight-bearing x-ray images, distal pancreatic guide plate assisted TKA can achieve accurate pancreas, obtain accurate lower extremity coronal and sagittal force lines, reduce blood loss, and improve recent pancreatic function [33, 34].

#### 3.2.3. Feature Processing and Analysis of Intelligent Electronic Medical CT Image

For the basic convolution operation in DNN, it naturally has the defect of paying too much attention to the calculation of local area in CT image of severe acute pancreatitis. In view of this defect, MS in amdrc net (multichannel aggregate spatial coding guided by long and short attention) greatly alleviates its deficiency. Compared with the general channel attention mechanism, the feature of long and short attention in this paper is that we use parallel channel attention and spatial attention and combine the feature graph conv4_ *X* is multiplied by the scaling coefficient obtained by the parallel attention module, and then the new feature graph conv4 after passing through the attention module is processed_ *X* by concat operation:

(21) $$\begin{array}{c} \theta \left(p,q\right)=\arctan\left(\frac{L\left(p,q+1\right)-L\left(p,q-1\right)}{L\left(p+1,q\right)-L\left(p-1,q\right)}\right). \end{array}$$

Then, the magnetic nanoparticles modified with EpCAM were used to capture sap, and then MUC1 aptamer was attached to the cell surface to form a Sandwich structure:

(22) $$\begin{array}{c} \ln\left(\frac{{\text{FI}}_{it}}{{\text{FI}}_{it}-1}\right)=\alpha +\beta \;\ln\;FI_{it}-1+\phi X_{it}-1+v_{i}+\tau_{t}, \end{array}$$

(23) $$\begin{array}{c} f\left(x\right)=\frac{1}{Nh}\sum_{i=1}^{N}k\left(\frac{X_{i}-x}{h}\right). \end{array}$$

The article "CT Image Changes of Severe Acute Pancreatitis Based on Smart Electronic Medical Augmented Reality in Nursing Practice" was retracted in 2023. Reasons: signs of a paper mill; suspected computer-generated content; unreliable results or conclusions; lack of ethics approval or compliance.

## 4. CT Image Changes of Severe Acute Pancreatitis in Nursing Practice

### 4.1. Pancreatitis and Immune Environment

As shown in Figure 1, the self-digestion process of pancreas during sap has an impact on the local inflammation and immune environment around it, resulting in the activation of a variety of inflammation and immune cytokines and local immune imbalance, resulting in abnormal pancreatic perfusion and decreased surfactant. Changes in pancreatic microcirculation cause diffuse edema of the pancreatic interstitium and pancreatic vesicles, damaging pancreatic lesions. Pathogenic infections of the intestine and the production of endotoxin can activate immune cells by invading pancreatic tissue and damage the capillaries and vesicles of the pancreas. In addition, the study also showed that the pancreatic injury in SAP patients was related to the changes of complement system and nuclear factor kB expression. The results showed that the incidence of pancreatic infection increased with the severity of SAP.

As shown in Table 1, the degree of pancreatic injury in patients with severe acute pancreatitis gradually aggravated with the extension of modeling time; drug can effectively improve the early condition of sap; with the progress of the disease, the expression of CARD9 mRNA and phosphorylated CARD9 protein in pancreatic tissue also increased; the expression and phosphorylation of CARD9 mRNA in pancreatic tissue of patients with severe acute pancreatitis in cqcqd group CARD9 protein was significantly lower than that of SAP group at the same time point.

As shown in Figure 2, patients with severe acute pancreatitis have severe neurological deficits and poor prognosis. The abnormal CT image in pancreas is related to the neurophysiological changes of pancreatic tissue during hypoperfusion. The decrease of neurovascular coupling and pancreatic blood flow in ischemic penumbra can increase slow wave activity and decrease fast wave activity. The decrease of pancreatic blood flow leads to the increase of low frequency wave activity, which is related to progressive neuronal death. Studies have shown that the abnormality of glutamate concentration (excitatory neurotransmitter) may be related to the CBF level of 20 ∼ 30 ml/(100gmin), and to the *δ* wave produced by the surviving neurons.

The article "CT Image Changes of Severe Acute Pancreatitis Based on Smart Electronic Medical Augmented Reality in Nursing Practice" was retracted in 2023. Reasons: signs of a paper mill; suspected computer-generated content; unreliable results or conclusions; lack of ethics approval or compliance.

As shown in Table 2, there were 21 cases of recurrence after internal drainage, and the cure rate was 91.1%. It is consistent with the literature reports. Internal drainage is an effective way to treat sap. Combined with the literature, the more the incidence of pancreatitis, the easier the recurrence of SAP after internal drainage, which may be related to repeated attacks of pancreatitis, repeated stimulation of inflammation, and pancreatic duct injury. On the other hand, 4 of the recurrent cases were SAP after chronic pancreatitis, and 50% of the recurrent cases were SAP after chronic pancreatitis. It may be related to chronic fibrosis of branch pancreatic duct and main pancreatic duct and continuous abnormal pancreatic drainage. Therefore, it is necessary to further explore the prognosis of SAP with different etiologies. In terms of complications, the overall complication rate was 16.6%, and one patient died of massive hemorrhage. Analysis of the causes of cyst recurrence and complications may be closely related to the mechanism of SAP development. The initiating factors of SAP are pancreatic tissue injury due to inflammation, trauma or microcirculation disturbance, and then pancreatic juice extravasation around the pancreas. It takes a certain time for the formation and strengthening of fibrous hoof tissue capsule wrapping pancreatic juice.

As shown in Table 3, early monitoring of regional blood flow changes and CT imaging abnormalities in ischemic lesions by QEEG and CT perfusion imaging can evaluate the neurological deficit of patients, which is also confirmed by the correlation between NIHSS score and various indicators in this paper. This paper analyzes the correlation between QEEG characteristics and CT perfusion imaging parameters, and the correlation between QEEG characteristics and NIHSS score. It is found that QEEG can be used as a reliable technical means to dynamically monitor the regional changes of ischemic lesions in SAP and can also dynamically assess the neurological deficit of patients in the early stage and timely guide the clinical adjustment of treatment strategies. However, due to the small sample size, this conclusion needs to be further demonstrated by increasing the sample size; in addition, due to the different types of CT imaging equipment, different parameter leads will affect the spatial specificity and accuracy of QEEG, and the parameters and algorithms of QEEG adopted by various manufacturers are also very different. In conclusion, there is a correlation between CT images and CTP features in SAP patients. Early dynamic monitoring of CT images can effectively evaluate the changes of ischemic focus and neuronal damage in patients.

The article "CT Image Changes of Severe Acute Pancreatitis Based on Smart Electronic Medical Augmented Reality in Nursing Practice" was retracted in 2023. Reasons: signs of a paper mill; suspected computer-generated content; unreliable results or conclusions; lack of ethics approval or compliance.

As shown in Figure 3, early pancreatic juice is highly irritant and inflammatory; the capsule of fibrous nodal tissue wrapping pancreatic juice is immature; early internal drainage and anastomosis are weak, and complications such as infection and recurrence are prone to occur. The experience of our center recommends that the time of surgical intervention should be extended as long as the patient's condition allows, rather than limited to 4–6 weeks.

As shown in Table 4, patients with asymptomatic SAP less than 6 cm were examined by abdominal color Doppler ultrasound every three months. Patients with cyst diameter more than 6 cm or less than 6 cm but with abdominal pain, pancreatic portal hypertension, and other symptoms were examined by abdominal enhanced CT. The size of pseudocyst, local symptoms, and endocrine and endocrine functions of patients were closely monitored, and disease progression was detected as soon as possible and appropriate intervention was given.

### 4.2. CT Image Analysis of Severe Acute Pancreatitis

As shown in Figure 4, if the course of disease is short and the cyst is small, but surgical treatment is necessary due to related symptoms, cyst gastric drainage is the first choice, because cyst gastric drainage can take an appropriate size opening on the gastric wall according to the size of the cyst, which can fully remove the necrotic tissue in the cyst, control inflammation as soon as possible, and reduce postoperative inflammatory edema. Gastric acid entering the cyst may have hemostatic and softening effects on the wound of the cyst wall. Postoperative placement of gastric tube in the cyst cavity and prone position can help to fully drain and promote the closure of the cyst cavity in a short time. However, Roux-en-Y drainage of cyst jejunum is not conducive to drainage due to the limited diameter of intestinal tube and the inaccessibility of gastric tube; and the increased number of Roux-en-Y anastomotic stoma also increases the risk of anastomotic leakage and stenosis. If the course of disease is long enough, the cyst tends to be mature and stable, and the thickness of the cyst is uniform and dense, the use of cyst stomach drainage or cyst jejunum (Roux-en-Y) drainage can achieve good results.

The article "CT Image Changes of Severe Acute Pancreatitis Based on Smart Electronic Medical Augmented Reality in Nursing Practice" was retracted in 2023. Reasons: signs of a paper mill; suspected computer-generated content; unreliable results or conclusions; lack of ethics approval or compliance.

As shown in Figure 5, clinicians should not only use targeted antibiotics according to the etiological results, but also pay attention to the infection prevention of patients during hospitalization, so as to avoid changing from noninfected patients to infected patients and increase the probability of adverse prognosis. The pathophysiological study of SAP mechanism has proved the important value of immune response for the disease. In the early stage of the disease, the cascade reaction of protease does not necessarily determine the severity of the disease. A variety of cytokines and complex inflammatory reactions are the basis of the pathogenesis and progress of SAP.

As shown in Figure 6, the current CT and MRI technology has provided great help for the diagnosis of pancreas, but studies have shown that neither CT nor MRI of craniopancreas can achieve real-time monitoring of regional changes of pancreatic ischemic lesions. CT imaging examination is relatively simple, and it can realize and dynamically observe the abnormal discharge of pancreas beside the bed. The traditional view is that QEEG has the advantage of real-time monitoring, but the spatial resolution is low, so it is not valuable to locate the lesion in pancreas. It can be seen from the figure that the abnormal *δ* wave of QEEG corresponds to the infarct center, while the *θ* wave and resting electrical activity are related to ischemic penumbra, pancreatic edema, and separation of nerve function. These findings confirm the value of QEEG in the localization of ischemic pancreas.

As shown in Figure 7, CT perfusion imaging has been used in clinical practice as a technique to accurately evaluate the hemodynamic changes of pancreas. In terms of pancreatic diagnosis, not only early detection of ischemic lesion areas but also real-time monitoring of hemodynamic changes in ischemic lesion areas is required, so CT perfusion imaging is particularly important. As shown in Table 5, there is a correlation between QEEG characteristics and CT perfusion imaging parameters in SAP patients. This conclusion can provide help in clinical diagnosis of SAP patients.

As shown in Figure 8, CT perfusion imaging can be used to observe the hemodynamic changes in different pancreatic regions, which can well determine the focus area. CT images are used to record the spontaneous formation of pancreatic biopotential. It is often used in the examination and diagnosis of epilepsy, pancreatitis, and intracranial space occupying lesions. The study found that when the blood flow of pancreatic tissue was interrupted for more than 3 seconds, the CT image showed abnormal changes in this area.

The article "CT Image Changes of Severe Acute Pancreatitis Based on Smart Electronic Medical Augmented Reality in Nursing Practice" was retracted in 2023. Reasons: signs of a paper mill; suspected computer-generated content; unreliable results or conclusions; lack of ethics approval or compliance.

As shown in Figure 9, due to the rapid progress of SAP patients in the early stage, CT image as a relatively simple means for dynamic monitoring is easier to achieve clinically, but there is still controversy about its monitoring effect at present. CT perfusion imaging has a good effect in evaluating the regional blood perfusion of ischemic lesions, but it cannot achieve real-time monitoring.

As shown in Table 6, the study of the correlation between QEEG characteristics and CT perfusion imaging has positive significance for the application of QEEG in dynamic monitoring of ischemic pancreas and guiding clinical treatment. The results showed that CBF was reduced, MTT and TTP were delayed, delta wave index, slow wave index, and BSI were increased, and ADR and dtabr were decreased in the ischemic lesion region compared to the contralateral region, CT perfusion imaging, and qEEG diagnostic values were further confirmed.

As shown in Figure 10, this paper analyzed the relationship between different pancreatic blood flow and qEEG and found that when the pancreatic blood flow was lower than 35 ml/(100g min), the fast beta rhythm disappeared, when the pancreatic blood flow was lower than 18 ML/(100g min), the delta rhythm began to appeared, and when the pancreatic blood flow was lower than 10 ml/(100g min), the CT image showed complete suppression. In the aspect of QEEG characteristics, the main indicators commonly used in the evaluation of ischemic pancreas are relative power ratio and BSI, among which ADR and dtabr are more commonly used, which are recognized as more accurate and stable evaluation and prediction indicators.

## 5. Conclusions

There are significantly more studies on CT image pancreatic guides in correcting coronal force lines than other plane force lines. Studies have shown that, compared with traditional TKA, CT imaging pancreas guide can better restore the coronal force line of the lower limbs, but there are also reports that there is no significant difference between the two. The results of this article show that the difference between postoperative mFTA and preoperative measurement is statistically significant and is similar to the mFTA result obtained by preparing CT image pancreatic guide plate combined with MRI and CT images of the whole lower limb. However, there was no statistically significant difference between FMAA and aLDFA and the preoperative measurement, indicating that the lower limb force line returned to the preoperative physiological state. We believe that a distal pancreatic guide plate created based on pancreatic CT and full-length x-ray images of the lower limbs can also improve the coronary force lines of the lower limbs. For fragile and severe acute pancreatitis caused by SAP, treatment should also be based on spleen deficiency.

The article "CT Image Changes of Severe Acute Pancreatitis Based on Smart Electronic Medical Augmented Reality in Nursing Practice" was retracted in 2023. Reasons: signs of a paper mill; suspected computer-generated content; unreliable results or conclusions; lack of ethics approval or compliance.

There are still some shortcomings in the syndrome rules of SAP secondary to severe acute pancreatitis discussed in this article. For example, under the guidance of TCM treatment theory, the inflammatory state of the pancreas can be improved in the early stage of SAP, thereby preventing or delaying the occurrence of glucose metabolism disorders. In addition, this article is the first to introduce CT images into the SAP model of patients with severe acute pancreatitis. Through chart analysis, it is found that the CARD9 mRNA expression level of the SAP model of severe acute pancreatitis is more sensitive, specific, and AUC than TNF-*α*, IL-1*β*, pathological scores. A high value indicates high diagnostic accuracy and can be used as a new target for assessing the state of SAP.

Due to the limited sample size in this article, individual differences in patients with severe acute pancreatitis may have an impact on the experimental results; the research team should also prepare pathological sections of multiple organs to observe the protective effect of drugs on multiple organs and at the same time continue to collect clinical trials in the future cases, a large sample size, multicenter clinical experimental research to verify the results of animal experiments. In summary, this article is the first to conduct a retrospective analysis of patients undergoing internal drainage treatment of SAP to explore the risk factors that affect the recurrence and complications of pseudocysts after internal drainage and provide clinical guidance.

## Figures and Tables

**Figure 1:** The self-digestion process of the pancreas during SAP.

**Figure 2:** Preparation of the patient's pancreas CT image (from Google: http://1il65.cn/tVz3ar).

**Figure 3:** Immature capsule of fibrous knot tissue encapsulating pancreatic juice.

**Figure 4:** The effect of SAP optosis-related protein compared with the early group (from Google: http://1il65.cn/tVz3ar).

**Figure 5:** Tumor cell-centered conversion to tumor growth microenvironment.

**Figure 6:** Important factors affecting DFS in patients undergoing radical surgery (from Google: http://1il65.cn/SsLUi3).

**Figure 7:** CT perfusion imaging as an accurate assessment.

**Figure 8:** Perfusion imaging to observe hemodynamic changes in different pancreatic regions.

**Figure 9:** Cancer manifestations of DS-8201 on HER2 expression (from Google: http://1il65.cn/SsLUi3).

**Figure 10:** The relationship between different pancreatic blood flow and QEEG.

The article "CT Image Changes of Severe Acute Pancreatitis Based on Smart Electronic Medical Augmented Reality in Nursing Practice" was retracted in 2023. Reasons: signs of a paper mill; suspected computer-generated content; unreliable results or conclusions; lack of ethics approval or compliance.

**Table 1:** Degree of pancreatic damage in patients with severe acute pancreatitis.

Item	Card9	Immune cells	SAP	SAP	MRI
SAP	1.09	3.5	1.69	1.12	3.9
Pancreas	3.88	3.77	3.88	3.39	4.04
Inflammation	2.89	2.07	4.93	1.25	3.42
Partial	4.8	3.14	3.58	3.29	4.14
Immune	5.72	3.08	2.09	4.02	3.19

**Table 2:** Number of occurrences of pancreatitis.

Item	Cells	SAP	SAP	MRI	SAP
SAP	0.33	1.44	1.35	1.41	0.44
Pancreas	3.9	2.9	3.66	2.89	2.49
Inflammation	4.04	2.14	5.46	2.67	2.61
Partial	3.42	1.04	1.54	1.25	5.07
Disorders	4.14	1.06	1.55	3.35	3.87
Card9	3.19	1.09	5.51	2.45	5.25

**Table 3:** QEEG and CT perfusion imaging to monitor ischemic lesions.

Item	SAP	Pancreas	Inflammation	Partial	Disorders
Cells	1.71	0.57	1.81	0.26	0.26
SAP	2.32	1.62	1.14	1.36	1.8
SAP	5.69	5.2	4.38	4.67	3.22
MRI	3.91	1.25	5.35	3.12	2
SAP	1.21	4.53	2.08	3.87	2.82

**Table 4:** Abdominal color Doppler ultrasound examination every 3 months.

Item	QEEG	CT perfusion	SAP	CPPE	mPFS	PPE
SAP	3.35	1.86	1.15	3.61	1.09	3.5
Pancreas	4.98	3.79	3.64	2.46	3.88	3.77
Inflammation	2.3	3.65	2.36	4.52	2.89	2.07
Partial	2.56	3.6	4.57	3.51	4.8	3.14
Disorders	5.69	6.87	3.82	3.47	5.72	3.08
Osimertinib	3.03	5.9	1.93	6.43	2.44	6.56

**Table 5:** QEEG characteristics and CT perfusion imaging parameters in SAP patients.

Item	SAP	Pancreas	Inflammation	Partial	Disorders
Cells	1.71	0.57	1.81	0.26	0.26
SAP	2.32	1.62	1.14	1.36	1.8
SAP	5.69	5.2	4.38	4.67	3.22
MRI	3.91	1.25	5.35	3.12	2
SAP	1.21	4.53	2.08	3.87	2.82

**Table 6:** Correlation between QEEG features and CT perfusion imaging.

Item	Epilepsy	Encephalitis	Intracranial	MRI	SAP
SAP	1.71	2.32	5.69	3.91	1.21
Pancreas	0.57	1.62	5.2	1.25	4.53
Inflammation	1.81	1.14	4.38	5.35	2.08
Partial	0.26	1.36	4.67	3.12	3.87
Disorders	0.26	1.8	3.22	2	2.82

## Data Availability

No data were used to support this study.
